The article "Genetic Diversity of Escherichia coli Coharboring mcr-1 and Extended Spectrum Beta-Lactamases from Poultry" was published in 2022. Journal: Biomed Res Int.

# Genetic Diversity of *Escherichia coli* Coharboring *mcr*-1 and Extended Spectrum Beta-Lactamases from Poultry

**DOI:** 10.1155/2022/8224883

**Published:** 2022-10-05

**Authors:** Arslan Jamil, Muhammad Asif Zahoor, Zeeshan Nawaz, Abu Baker Siddique, Mohsin Khurshid

**Affiliations:** Department of Microbiology, Government College University Faisalabad, Pakistan

## Abstract

**Background:**

The emergence of resistance to beta-lactam agents in poultry results in multidrug-resistant (MDR) phenotypes in *Escherichia coli* isolates from poultry birds. The appearance of mobile colistin resistance (*mcr*) genes in the poultry sector has further worsened the situation. Therefore, the current study is aimed at investigating the molecular epidemiology of *mcr* harboring colistin-resistant *E. coli* among poultry.

**Methods:**

The isolation and identification of colistin-resistant *E. coli* (CR-Ec) were done from the broiler's fecal samples through culturing using selective media supplemented with colistin sulfate (4 *μ*g/ml). The antibiogram studies of the isolates were performed using the disc diffusion method and broth microdilution method as per CLSI guidelines. The screening for the genes conferring resistance to colistin as well as beta-lactam agents was performed by PCR. The genetic diversity of *mcr-*positive strains was assessed by multilocus sequencing typing (MLST).

**Results:**

Out of 500 fecal samples, 7% (35/500) were found positive for the presence of colistin-resistant *E. coli* (CR-Ec). Among the CR-Ec isolates, 74.28% (26/35) were detected as ESBL producers carrying the *bla*CTX-M-1 gene in 15/35 (42.85%) isolates and *bla*CTX-M-15 and *bla*TEM genes in 21/35 (60%) and 35/35 (100%) isolates, respectively. *E. coli* isolates were found positive for the presence of *mcr*-1, although none of the isolates exhibited the *mcr*-2 or *mcr*-3 genes. The MLST of CR-Ec has shown the ST1035 as the most prevalent genotype, while 82.85% (29/35) of CR-Ec strains belonged to clonal complex (CC) 131 comprising ST1035, ST131, ST1215, ST1650, and ST2279.

**Conclusions:**

The findings suggest a continuous monitoring system in veterinary and clinical settings to avoid unnecessary antibiotics. Further studies are needed at the national level to help control the increasing resistance among Enterobacterales in poultry settings.

## 1. Introduction

*Escherichia coli* is an emerging pathogen that is associated with multiple infections in humans such as urinary tract infection (UTI), bacteremia, meningitis, and travelers' diarrhea [1]. Similarly, *E. coli* is also responsible to cause colibacilloses among animals. It is the most adaptable microorganism with multiple pathogenic strains among humans and animals that causes a variety of infections. In the case of poultry, *E. coli* is responsible for respiratory tract infections such as colibacillosis through the inhalation of fecal contaminated dust [2]. *Escherichia coli* strains isolated from commercial broilers are frequently resistant to antibiotics [3]. Numerous studies have indicated that improper use of antimicrobial agents in food animals including poultry leads to the emergence of antimicrobial-resistant strains [4]. The infections among the animals caused by *E. coli* are treated with the various routinely used antibiotics such as streptomycin, sulfonamide, colistin, ampicillin, polymyxins, cephalosporins, fluoroquinolones, and tetracycline, depending upon the type and nature of infection [5].

Extended-spectrum beta-lactamases (ESBLs) are a group of enzymes that frequently confer resistance against beta-lactam drugs such as third-generation cephalosporins, i.e., cefotaxime, ceftazidime, and ceftriaxone [6–8]. The ESBLs are derived from narrow-spectrum beta-lactamase genes such as TEM-1, TEM-2, or SHV-1 that have undergone mutations altering the amino acid types and configurations, especially around the active site of the enzyme. They are usually encoded by the plasmids, and therefore, are readily exchanged between the bacterial species. Thus far, more than 350 ESBL variants have been reported commonly among the members of the Enterobacteriaceae family mainly *Escherichia coli* and *Klebsiella pneumoniae* [9].

Colistin belongs to the polymyxin group of drugs that were considered a drug of last resort for the therapeutic management of infections caused by MDR *Enterobacteriaceae* family members such as *E. coli*. Colistin-resistant bacteria are worldwide important as they pose a major threat to public and animal health [8, 10]. After the first report of *mcr*-1, numerous mobile colistin resistance variants have been reported across many countries in the five continents. So far, 10 different *mcr* genes and their several variants have been reported from various parts of the world from different bacterial isolates, from the environment, animals, humans, food, and poultry farms [11, 12]. In Pakistan, the studies have reported *mcr*-1 and *mcr*-2 only. The *mcr*-1 was reported in *E. coli* isolates from humans, broilers, and wildlife in Pakistan [13–15]. In a recent study, a total of 250 fecal samples were collected from poultry and livestock, and 153 strains of *E. coli* were recovered of which 49.01% were carrying the ESBL genes and 18.95% colistin-resistant harboring *mcr*-1 gene [16]. In a study from the clinical settings in Pakistan, 545 *E. coli* strains were obtained from the clinical samples, and only four (0.73%) were resistant to colistin and carrying *mcr-1* [17].

Therefore, the current study was designed to investigate the prevalence, characterization, and genetic diversity of colistin resistance *E. coli* (CR-Ec) isolated from fecal samples of commercial broilers that were harboring extended-spectrum beta-lactamases (ESBLs) and mobile colistin-resistant (*mcr*-1) genes.

## 2. Materials and Methods

### 2.1. Ethical Approval

The study was approved by the institutional review board (Government College University Faisalabad, Pakistan) before the isolation of bacterial strains and collection of the data.

### 2.2. Isolation of Colistin-Resistant *Escherichia coli*

500 fecal samples were collected from the commercial broiler from five different farms located in Faisalabad, Pakistan. All samples were collected using the sterile spatula and transferred to 50 ml sterile tubes and were shifted to the laboratory immediately for initial processing. The samples were first processed on MacConkey agar and Eosin Methylene Blue agar (Oxoid™ UK) supplemented with colistin sulfate (4 *μ*g/ml) and incubated at 37°C for 24 hours. Moreover, additional confirmation, as well as precise identification of all isolates, was done through various biochemical tests including citrate utilization test, Voges-Proskauer test, indole formation, motility test, carbohydrate fermentation test, hydrogen sulfide production, catalase, oxidase, and urease tests, and methyl red tests followed by confirmation by API 20E (BioMerieux, France).

### 2.3. Molecular Identification of *Escherichia coli*

The extracted genomic DNA was investigated through polymerase chain reaction by using the species-specific primer (*uidA*) gene set (listed in Table 1) amplification conditions as initial denaturation (95°C for 03 minutes), 35 cycles of denaturation (95°C for 30 seconds), annealing (58°C for 30 seconds), the cyclic extension (72°C for 01 minute), as well as a final extension at 72°C for 10 minutes using the thermocycler (T100™ Thermal Cycler, Bio-Rad).

### 2.4. Antibiotic Susceptibility Test (AST)

Antibiotic susceptibility testing of isolates was performed using the disc diffusion method according to the Clinical and Laboratory Standard Institute Guideline (CLSI) (2022) to evaluate the antibacterial activity against the different antimicrobial agents which were all obtained from Oxoid (UK) such as amikacin (30 *μ*g), gentamicin (10 *μ*g), tobramycin (10 *μ*g), ciprofloxacin (5 *μ*g), ceftazidime (30 *μ*g) cefepime (30 *μ*g), cefotaxime (30 *μ*g), amoxycillin/clavulanic acid (30 *μ*g), ampicillin/sulbactam (20 *μ*g), piperacillin/tazobactam (110 *μ*g), imipenem (10 *μ*g), meropenem (10 *μ*g), trimethoprim/sulfamethoxazole (25 *μ*g), tetracycline (30 *μ*g), and doxycycline (30 *μ*g).

Using the broth microdilution method, minimum inhibitory concentration (MIC) of *E. coli* strains against several antimicrobials was performed including amikacin, gentamicin, tobramycin, ciprofloxacin, cefotaxime, ceftazidime, cefepime, imipenem, meropenem, colistin, as well as tigecycline. The results were interpreted according to CLSI (2022) guidelines. *Escherichia coli* (ATCC-25922) was used as a quality control strain for the susceptibility profiling.

### 2.5. Detection of ESBL and *mcr* Genes

The extracted bacterial genomic DNA was subjected to a polymerase chain reaction for screening of ESBL genes using the primers for different ESBL encoding genes conferring resistance such as *bla*_CTX-M_*, bla*_CTX-M-1_, *bla*_CTX-M-2_, *bla*_CTX-M-8_, *bla*_CTX-M-9_, *bla*_CTX-M-10_, *bla*_CTX-M-14_, *bla*_CTX-M-15_, *bla*_SHV_, and *bla*_TEM_ genes as well as colistin resistance genes (*mcr*-1, *mcr*-2, and *mcr*-3). The PCR was run on the Thermal Cycler (T100™, Bio-Rad, USA). The conditions for PCR were as follows: initial denaturation at 94°C for 3 minutes, cyclic denaturation at 94°C for 1 minute, annealing temperature (variable, Table 1) for 45 seconds, cyclic extension at 72°C for 1 minute, and final extension at 72°C for 7 minutes. The PCR data including sets of primer sequence, annealing temperature, and product size (bp) are mentioned in Table 1. Afterward, the amplified PCR product was subjected to Sanger sequencing (Macrogen, South Korea). The obtained sequence data was compared using the BLAST tool.

### 2.6. Multilocus Sequence Typing (MLST)

All *mcr*-1-positive stains were subjected to multilocus sequencing typing (MLST). According to the conditions described by Entero-base Database, the Achtman 7 Gene (MLST) was performed through the amplification of seven housekeeping genes as *adK*, *fumC*, *gyrB*, *icd*, *mdh*, *purA*, and *recA* as described previously [18]. Agarose gel PCR amplicons were extracted through the GeneJet Gel Extraction Kit (Thermo Scientific™) and were sequenced by Macrogen, South Korea. After initial editing from the ChromasPro (Technelysium, Australia), these sequences were aligned from the ClustalW Algorithm (MEGA software), whereas allelic numbers were assigned to each gene loci. The Entero-base Database was accessed to find the allelic profiles of isolates and to know the sequencing types (STs).

## 3. Results

### 3.1. Occurrence of *E. coli*

A total of 35 (7%) fecal samples were positive for the CR-Ec. The *E. coli* were identified by biochemical methods and further confirmed by the amplification of the *uid*A gene.

### 3.2. Antibiotic Susceptibility

The CR-Ec isolates were tested against the different antibiotics and showed variable resistance profiles. The 91.4% isolates were resistant to gentamicin (CN), 88.6% to tetracycline (TE), 74.3% to cefepime (FEP), ceftazidime (CAZ), cefotaxime, amoxicillin/clavulanic acid (AMC) and piperacillin/tazobactam, 71.4% to ampicillin/sulbactam (SAM), 68.6% to ciprofloxacin (CIP), 62.9% to amikacin (AK) and doxycycline (DO), 60% to sulfamethoxazole/trimethoprim (SXT), and 31.4% to tobramycin (TOB). However, all isolates were found 100% susceptible to imipenem (IMP), meropenem (MEM), and tigecycline (TGC). The MIC results have shown that the MIC values for CR-Ec isolates varied from 4 to 16 *μ*g/ml against colistin as shown in Table 2.

### 3.3. Detection of ESBL Genes

The CR-Ec isolates were screened for the ESBL genes (*bla*_CTX-M_, *bla*_CTX-M-1_, *bla*_CTX-M-2_, *bla*_CTX-M-8_, *bla*_CTX-M-9_, *bla*_CTX-M-10_, *bla*_CTX-M-14_, and *bla*_CTX-M-15_ as well as *bla*_SHV_ and *bla*_TEM_ genes) using polymerase chain reaction. PCR results exhibited that 74.28% (26/35) isolates were found to harbor the ESBL genes. The bla_CTX-M-1_ was found in 42.85% (15/35) of CR-Ec isolates whereas both *bla*_CTX-M-15_ and *bla*_TEM_ were found in 60% (21/35) of CR-Ec isolates (Table 3).

### 3.4. Mobile Colistin-Resistant Genes (*mcr*-1) Screening

The 35 CR-Ec isolates that were phenotypically confirmed were subjected to PCR for screening of *mcr*-1, *mcr*-2, and *mcr*-3 genes. PCR investigation confirmed that all of these isolates were positive for the presence of *mcr*-1, and none of the isolates were found positive for the *mcr*-2, or *mcr*-3 genes (Table 3).

### 3.5. Multilocus Sequence Typing (MLST)

Multilocus sequence typing (MLST) has shown that *E. coli* belongs to multiple sequence types. ST1035 (*n* = 11, 31.4%) was found to be the most prevalent genotype, which was detected among 11 *E. coli* isolates, and eight CR-Ec isolates (*n* = 8, 22.8%) corresponding to ST131 that was harboring *mcr*-1 and ESBLs. Similarly, ST1215 corresponded to 5 (14.8%) isolates, whereas 4 (11.4%) isolates belonged to ST2279 and ST88. The ST1650 accounted for 3 (8.5%) isolates. Each ST410, ST10, ST23, and ST3059 corresponded to (2.8%) isolates. Of the 35 colistin-resistant *E. coli* (CR-Ec) strains, 82.85% (29/35) isolates belong to clonal complex (CC) 131 comprising ST1035, ST131, ST1215, ST1650, and ST2279 (Table 3).

## 4. Discussion

Globally, antimicrobial resistance is a serious issue, but in developing countries, the excessive use of antimicrobials in veterinary settings has made the situation, even more, worse [4, 19]. In Pakistan, colistin is used extensively to treat colibacillosis and clostridial enteritis in poultry, either alone or in combination with other antibiotics [20]. The emergence of *mcr* genes among poultry-origin bacterial isolates and colistin resistance is directly related to the increased use of colistin [21]. Hence, the current study was designed to describe the genetic diversity of CR-Ec strains isolated from the fecal samples of commercial broilers and to find out the prevalence of ESBL and mobile colistin resistance genes.

In this study, 500 fecal samples were screened for CR-Ec and obtained 35 isolates and all of them harbored the *mcr*-1 gene. The comparison with some past studies has shown the variation among colistin resistance phenotypes in poultry samples. Recently, in a study from Egypt, 56 *E. coli* isolates were obtained from 120 poultry specimens, and 25% (14/56) isolates were positive for the *mcr* genes [22]. The incidence rate of colistin resistance among poultry birds was reported as 6.6% in Bangladesh [23]. In a study from China, the rate of colistin resistance among *E. coli* isolates from poultry farms increased from 4.1% (2014) to 16.2% (2019) [24].

The antibiotic susceptibility profiling of CR-Ec showed variable resistance to antibiotics such as gentamicin (91.4%), tetracycline (88.6%), cefepime, ceftazidime, cefotaxime, amoxicillin/clavulanic acid, and piperacillin/tazobactam (74.3%), ampicillin/sulbactam (71.4%), ciprofloxacin (68.6%), amikacin and doxycycline (62.9%), sulfamethoxazole/trimethoprim (60%), and tobramycin (31.4%) (Figure 1). All isolates were found susceptible to imipenem, meropenem, and tigecycline. As the previous study from Pakistan, 98% of *E. coli* isolates were resistant to ampicillin, 95% to tetracycline, 72% to ciprofloxacin, 69% to colistin, 68% to chloramphenicol, 67% to sulfamethoxazole/trimethoprim, and 27% to cefotaxime, whereas all isolates were found susceptible to imipenem [25]. A study from Tunisia have reported that *E. coli* strains from poultry were found resistant against nalidixic acid (92%), flumequine (86%), doxycycline (82%), amoxicillin (78%), tetracycline (76%), amoxicillin/clavulanic (74%), enrofloxacin (68%), cefotaxime (68%), ceftazidime (66%), aztreonam (62%), cefepime (58%), and colistin (24%), respectively [26].

In the current study, the MIC values of CR-Ec isolates for colistin ranged from 4 to 16 *μ*g/ml. However, all colistin-resistant isolates were susceptible to imipenem, meropenem (MIC < 4 *μ*g/ml), and tigecycline (MIC < 8 *μ*g/ml).

The present study has evaluated the prevalence of ESBL genes among CR-Ec isolates from poultry fecal samples. A total of 74.28% (26/35) CE-Ec isolates were screened positive for ESBL genes (Table 3). The screening for ESBL genes has shown that *bla*_CTX-M_ was the major ESBL genotype. The *bla*_CTX-M1_ was found in 42.85% (15/35), whereas 60% (21/35) of isolates were carrying the *bla*_CTX-M15_ and *bla*_TEM_ genes (Table 3). A systematic review has described the data of 1329 *E. coli* strains, and the *bla*_CTX-M_ and *bla*_TEM_ were the common ESBL families in humans and 70 chicken-originating isolates [27]. The study has shown that ESBLs carrying *E. coli* from poultry birds carry multiple types of beta-lactamase genes, but the predominant combination was *bla*_CTX_ and *bla*_TEM_ [28]. This difference in the prevalence of ESBL gene could be due to specimen type and its processing, geographical changes, flock size as well as local practices for antibiotics use [29].

This study also screened for the incidence of *mcr*-1, *mcr*-2, and *mcr*-3 genes among colistin-resistant *E. coli* (CR-Ec) and found that 100% (35/35) of isolates were positive for *mcr*-1, and none of the isolates were found positive for *mcr*-2 and *mcr*-3 gene (Table 3). In contrast, comparable studies in Nepal and Iran reported that the *mcr*-1 gene is less prevalent among poultry-origin CR-Ec strains [30–32]. However, identical studies conducted in Bangladesh and Denmark published a similar prevalence of the *mcr*-1 gene among ESBLs producing CR-Ec [33]. The study is identical to a study from Egypt that reported a 100% prevalence of the *mcr*-1 gene, whereas *mcr*-2, *mcr*-3, *mcr*-4, and *mcr*-5 genes were not found in any of the isolates [22]. In addition, similar findings with the presence of the *mcr*-1 gene only were published in Morocco, North Africa, Algeria, Tunisia, and many other countries [34, 35]. An investigation of chicken birds in Faisalabad, Pakistan, found that 8 out of 100 *E. coli* isolates were positive for *mcr*-1 [21]. Our results strongly agreed with various previous reports suggesting that *mcr*-1 is the most important and widespread gene among CR-Ec isolates from poultry [36].

The multilocus sequence type (MLST) analysis of CR-Ec has shown that the strains belong to various sequence types (STs). A total of thirty-five *E. coli* isolates were characterized by MLST, and 10 different STs were observed. Among the STs, the most prevalent sequence types are ST1035, ST131, ST1215, ST1650, and ST2279 which belong to clonal complexes (CC) 131 while other sequence types including ST410, ST88, ST23, and ST88 belonged to the clonal complexes 23 (CC). One isolate belonging to ST10 corresponded to clonal complex 10 (CC) as shown in Table 3. A study from China reported ST10 from clinical samples [37]. The ST10 sequence type was well known for being prevalent in food and human stool samples [38]. Previous reports have indicated that poultry harboring the *mcr* gene belonged to ST410 [39], ST156, and ST641 [40, 41]. In this study, there was one strain of *E. coli* belonging to ST410 harboring *mcr*-1. This ST410 strain represents its widespread distribution around the globe, has been previously reported from North America, Europe, South America, Asia, and Africa, and was indicating its ability to survive for a long time in a specific host [42]. Our findings disclosed that the majority, i.e., twenty-nine isolates, belonged to CC131. As far as the ST131 is concerned, it usually carries the ESBLs and contains *bla*CTX-M-15 in the majority of cases [43]. Moreover, ST131 was also found to harbor the *mcr*-1 gene and isolated among the chicken birds in various European countries including France, Germany, Hungary, Spain, and the United Kingdom [44]. In the present study, ST23 was reported in one isolate which harbored *mcr*-1. The ST23 was previously reported by China which harbored ESBL-resistant genes including *bla*_CTX-M_, *bla*_TEM_, and *bla*_SHV_ [45]. Generally, it is fact that *mcr* genes have been identified on diverse STs in *E. coli* isolated from human, animal, and food samples suggesting the dissemination of genes successfully through the mobile genetic element (MGE) and plasmid rather than dissemination of specific clones of *E. coli* [46].

The scientific interests have inclined toward the transmissible colistin resistance (mcr) mediated by the plasmids since their discovery in 2015 as plasmid-mediated resistance can more readily disseminate among the Enterobacterales compared to the chromosomal-mediated resistance, especially in the livestock sector. It is assumed that with the reduction in the consumption of colistin in veterinary medicine, the prevalence of the *mcr* gene harboring plasmids could reduce due to the absence of selective pressure of colistin. In contrast, the Enterobacterales isolates from humans mostly resist colistin due to chromosomal mutations, and their prevalence will keep on increasing as colistin is increasingly being used as a drug of last resort for the therapeutic management of infections caused by the carbapenemase-producing pathogens [47]. The systematic review of literature from high-income countries also indicates that ST10, ST88, ST410, and ST131 are commonly reported in *E. coli* isolates from poultry [48]. The current study highlighted the emergence of *mcr*-1 harboring *E. coli* in the poultry sector in Pakistan which poses a significant threat to public health. It is a need of the hour to monitor and control the use of antibiotics especially colistin in the poultry sector. Moreover, future studies are needed to screen for such resistant determinants on a larger scale.

## 5. Conclusion

The current study has reported the genetic diversity among CR-Ec isolates harboring *mcr*-1 and ESBLs from commercial broilers from Pakistan. The presence of *mcr*-1 in all of CR-Ec isolates associated with the clonal complex (CC) 131 is alarming as this clonal complex is also associated with a higher number of infections in clinical settings. Pakistan is the one of top poultry producers in Asia; therefore, the research should be widely extended toward the screening of MDR bacterial species in poultry to avoid any epidemic caused by such MDR pathogens. It is highly recommended to closely monitor the colistin and beta-lactam-resistant *E. coli* strains in veterinary and clinical settings.

## Figures and Tables

**Figure 1:** Antimicrobial susceptibility pattern of colistin-resistant *Escherichia coli* from poultry.

**Table 1:** PCR primers list for amplifications of resistance genes determinates.

Target gene name	Primers (name)	Sequences	Annealing (temperature)	Product
*uid*A	(uid-A)-(F) (uid-A)-(R)	CAACGAACTGAACTGGCAGA CATTACGCTGCGATGGAT	58	162
*bla*_CTX-M_	CTX-MU-(F) CTX-MU-(R)	ATGTGCAGYACCAGTAARGT TGGGTRAARTARGTSACCAGA	52	593
*bla*_CTX-M-1_	CTX-M-1-(F) CTX-M-1-(R)	GGTTAAAAAATCACTGCGTC TTACAAACCGTYGGTGACGA	50	873
*bla*_CTX-M-2_	CTX-M-2-(F) CTX-M-2-(R)	ATGATGACTCACAGCATTCG TCCCGACGGCTTTCCGCGTT	56	833
*bla*_CTX-M-8_	CTX-M-8-(F) CTX-M-8-(R)	TTTGCCCGTGCGATTGG CGACTTTCTGCCTTCTGCTCT	50	368
*bla*_CTX-M-9_	CTX-M-9-(F) CTX-M-9-(R)	ATGGTGACAAAGAGAGTGCA CCCTTCGGCGATGATTCTC	50	870
*bla*_CTX-M-10_	CTX-M-10-(F) CTX-M-10-(R)	GCAGCACCAGTAAAGTGATGG GCGATATCGTTGGTGGTACC	56	524
*bla*_CTX-M-14_	CTX-M-14-(F) CTX-M-14-(R)	GAGAGTGCAACGGATGATG TGCGGCTGGGTAAAATAG	56	941
*bla*_CTX-M-15_	CTX-M-15-(F) CTX-M-15-(R)	CACACGTGGAATTTAGGGACT GCCGTCTAAGGCGATAAACA	50	995
*bla*_TEM_	TEM-(F) TEM-(R)	TTGGGTGCACGAGTGGGTTA TAATTGTTGCCGGGAAGCTA	55	506
*bla*_SHV_	SHV-(F) SHV-(R)	ATGCGTTATATTCGCCTGTG AGATAAATCACCACAATGCGC	56	896
*mcr*-1	*mcr*-1-(F) *mcr*-1-(R)	AGTCCGTTTGTTCTTGTGGC AGATCCTTGGTCTCGGCTTG	60	320
*mcr*-2	*mcr*-2-(F) *mcr*-2-(R)	AGCCGAGTCTAAGGACTTGATGAATTTG GCGGTATCGACATCATAGTCATCTTG	57	576
*mcr*-3	*mcr*-3-(F) *mcr*-3-(R)	CGCTTATGTTCTTTTTGGCACTGTATT TGAGCAATTTCACTATCGAGGTCTTG-3	57	1067

**Table 2:** Minimum inhibitory concentration distribution of colistin-resistant *Escherichia coli* isolates.

Antimicrobial agents	Breakpoints	No. of isolates with MIC (*μ*g/ml) of										
		≤0.25	0.5	1	2	4	8	16	32	64	128	≥256
Amikacin	≥64	—	—	—	6	4	3	—	—	4	11	7
Gentamicin	≥16	—	—	2	1	—	—	1	12	11	7	1
Tobramycin	≥16	—	—	8	13	2	—	1	6	2	3	—
Ciprofloxacin	≥1	11	—	—	—	—	2	12	5	4	1	—
Cefotaxime	≥4	2	6	1	—	—	1	9	12	3	1	—
Ceftazidime	≥16	—	1	7	1	—	—	—	2	16	7	1
Cefepime	≥16	2	3	4	—	—	—	2	6	15	3	—
Imipenem	≥4	25	10	—	—	—	—	—	—	—	—	—
Meropenem	≥4	20	11	4	—	—	—	—	—	—	—	—
Colistin	≥4	—	—	—	—	20	14	1	—	—	—	—
Tigecycline	≥8	13	19	3	—	—	—	—	—	—	—	—

**Table 3:** Sequence types of *Escherichia coli* isolates harboring ESBL and *mcr* genes.

Isolate	ST	CC	MIC of antimicrobial agents												ESBL and colistin-resistant determinants
			AK	CN	TOB	CIP	CTX	CAZ	FEP	IMP	MEM	CT	SXT	TGC	
CR-Ec1	131	ST131 Cplx	128	32	32	16	16	64	32	0.25	0.25	8	32	0.5	bla_CTX-M-1_, *bla*_CTX-M-15_, *bla*_TEM_, *mcr*-1
CR-Ec2	1035	ST131 Cplx	128	128	4	16	32	64	64	0.25	0.25	4	8	0.5	*bla*_CTX-M-15_, *bla*_TEM_, *mcr*-1
CR-Ec3	131	ST131 Cplx	256	64	32	32	16	128	16	0.5	0.5	8	32	0.5	bla_CTX-M-1_, *bla*_CTX-M-15_, *bla*_TEM_, *mcr*-1
CR-Ec4	131	ST131 Cplx	128	32	32	16	32	64	32	0.25	0.25	8	32	0.25	bla_CTX-M-1_, *bla*_CTX-M-15_, *bla*_TEM_, *mcr*-1
CR-Ec5	1215	ST131 Cplx	8	64	2	16	16	64	64	0.5	0.5	4	0.5	0.5	bla_CTX-M-1_, *mcr*-1
CR-Ec6	1035	ST131 Cplx	256	32	2	8	32	64	64	0.25	0.5	4	8	1	*bla*_CTX-M-15_, *bla*_TEM_, *mcr*-1
CR-Ec7	131	ST131 Cplx	256	64	128	16	16	64	64	0.25	0.25	8	16	0.5	bla_CTX-M-1_, *bla*_CTX-M-15_, *bla*_TEM_, *mcr*-1
CR-Ec8	1035	ST131 Cplx	128	32	2	32	64	128	64	0.25	0.25	8	8	0.25	*bla*_CTX-M-15_, *bla*_TEM_, *mcr*-1
CR-Ec9	131	ST131 Cplx	256	128	64	64	64	256	128	0.25	0.25	16	32	0.25	bla_CTX-M-1_, *bla*_CTX-M-15_, *bla*_TEM_, *mcr*-1
CR-Ec10	1650	ST131 Cplx	4	32	2	0.25	0.5	1	1	0.25	0.25	4	0.25	0.5	*mcr*-1
CR-Ec11	1035	ST131 Cplx	64	16	1	8	32	64	64	0.25	0.25	4	8	0.5	*bla*_CTX-M-15_, *bla*_TEM_, *mcr*-1
CR-Ec12	1035	ST131 Cplx	128	32	2	16	32	128	128	0.5	0.5	4	8	1	*bla*_CTX-M-15_, *bla*_TEM_, *mcr*-1
CR-Ec13	1035	ST131 Cplx	64	32	1	16	32	64	64	0.5	0.5	4	8	0.5	*bla*_CTX-M-15_, *bla*_TEM_, *mcr*-1
CR-Ec14	131	ST131 Cplx	128	32	64	16	32	64	64	0.25	0.5	8	32	0.25	bla_CTX-M-1_, *bla*_CTX-M-15_, *bla*_TEM_, *mcr*-1
CR-Ec15	1215	ST131 Cplx	2	128	1	32	16	64	64	0.25	0.25	8	0.5	0.5	bla_CTX-M-1_, *mcr*-1
CR-Ec16	2279	ST131 Cplx	128	64	32	0.25	32	64	64	0.5	1	8	8	0.5	bla_CTX-M-1_, *bla*_CTX-M-15_, *bla*_TEM_, *mcr*-1
CR-Ec17	131	ST131 Cplx	256	64	16	64	16	64	16	0.25	0.25	8	32	0.5	bla_CTX-M-1_, *bla*_CTX-M-15_, *bla*_TEM_, *mcr*-1
CR-Ec18	1650	ST131 Cplx	2	64	2	0.25	1	0.5	1	0.25	0.25	4	0.5	1	*mcr*-1
CR-Ec19	410	ST23 Cplx	2	256	128	0.25	0.5	1	0.5	0.25	0.5	4	0.5	0.25	*mcr*-1
CR-Ec20	1035	ST131 Cplx	128	64	2	64	16	64	32	0.5	0.5	4	16	0.5	*bla*_CTX-M-15_, *bla*_TEM_, *mcr*-1
CR-Ec21	1035	ST131 Cplx	64	32	1	16	64	128	128	0.25	0.25	4	8	0.25	*bla*_CTX-M-15_, *bla*_TEM_, *mcr*-1
CR-Ec22	1035	ST131 Cplx	128	128	4	32	32	64	64	0.25	0.25	4	8	0.5	*bla*_CTX-M-15_, *bla*_TEM_, *mcr*-1
CR-Ec23	1035	ST131 Cplx	64	32	1	16	128	128	64	0.25	0.25	4	16	0.25	*bla*_CTX-M-15_, *bla*_TEM_, *mcr*-1
CR-Ec24	1215	ST131 Cplx	8	128	2	16	16	32	32	0.5	1	8	0.25	0.5	bla_CTX-M-1_, *mcr*-1
CR-Ec25	131	ST131 Cplx	256	128	32	128	32	128	32	0.25	0.25	8	32	0.5	bla_CTX-M-1_, *bla*_CTX-M-15_, *bla*_TEM_, *mcr*-1
CR-Ec26	2279	ST131 Cplx	128	128	128	0.25	32	128	64	0.25	0.25	8	8	0.25	bla_CTX-M-1_, *bla*_CTX-M-15_, *bla*_TEM_, *mcr*-1
CR-Ec27	1650	ST131 Cplx	8	64	1	0.25	0.25	1	0.25	0.25	0.5	4	0.25	0.25	*mcr*-1
CR-Ec28	88	ST23 Cplx	2	1	2	0.25	0.5	2	1	0.5	1	4	0.5	0.5	*mcr*-1
CR-Ec29	10	ST10 Cplx	128	64	32	0.25	0.5	1	0.5	0.25	0.25	4	0.5	0.25	*mcr*-1
CR-Ec30	23	ST23 Cplx	4	32	2	0.25	0.25	1	0.25	0.25	0.25	8	1	0.25	*mcr*-1
CR-Ec31	1215	ST131 Cplx	4	64	1	32	16	64	64	0.5	0.5	4	0.5	0.25	bla_CTX-M-1_, *mcr*-1
CR-Ec32	1215	ST131 Cplx	2	32	1	16	8	32	32	0.5	1	4	0.5	0.25	bla_CTX-M-1_, *mcr*-1
CR-Ec33	1035	ST131 Cplx	256	64	2	64	32	64	64	0.25	0.25	4	8	0.5	*bla*_CTX-M-15_, *bla*_TEM_, *mcr*-1
CR-Ec34	88	ST23 Cplx	4	2	2	0.25	0.5	1	1	0.25	0.5	4	1	0.5	*mcr*-1
CR-Ec35	3059	—	2	1	2	0.25	0.5	1	0.5	0.25	0.25	8	0.5	0.5	*mcr*-1

*MCR*-1, ESBLs, and clonal complex (CC).

## Data Availability

All data used to support the findings of this study are included in the article.
